The article "Study on Antidepressant Emotion Regulation Based on Feedback Analysis of Music Therapy with Brain-Computer Interface" was published in 2022. Journal: Comput Math Methods Med.

# Study on Antidepressant Emotion Regulation Based on Feedback Analysis of Music Therapy with Brain-Computer Interface

**DOI:** 10.1155/2022/7200678

**Published:** 2022-10-05

**Authors:** Mengru Sun

**Affiliations:** School of Sookmyung Women's University, Seoul 04310, Republic of Korea

## Abstract

In today's society, people with poor mental ability are prone to neuropsychiatric diseases such as anxiety, ADHD, and depression due to long-term negative emotions. Although conventional Western medicine has certain curative effect, these drugs have significant anticholinergic side effects central toxicity as well as cardiovascular and gastrointestinal side effects which limit their application in the elderly. At present, several antidepressants used in clinic have certain limitations. According to the symptoms of depression, this paper proposes a feedback emotion regulation method of brain-computer interface music therapy. This method uses special music stimulation to regulate the release of inhibiting sex hormones in the body, reduce the influence of negative emotions on the internal environment of the body, and maintain the steady state of the body. In this method, EEG is used as the emotional control signal of depressed patients, and this biological signal is transformed into music that depressed patients can understand, so as to clarify their physiological and psychological state and realize emotional self-regulation by feedback.

## 1. Introduction

In this review, music therapy is examined as evidence of a treatment. To evaluate the effect of music therapy on behavioral, social, cognitive, and emotional problems in Alzheimer's patients, a randomized controlled trial was conducted to report the clinical outcomes of music therapy for behavioral, social, cognitive, and emotional problems in Alzheimer's patients [1]. Music, as a specific stimulus, combines motion and stimulation through different sensory pathways to obtain motor and emotional responses. In this study, a prospective, randomized, controlled, and single blind method was used to study the effects of music therapy on motor and emotional function of Parkinson's patients. MT is effective for motor, emotional, and behavioral functions. We propose active MT as a new method to be included in PD rehabilitation program [2]. Many studies have shown that listening to music activates many brain structures involved in cognition, sensorimotor, and emotional processing. This paper briefly summarizes the factors affecting the effect of music therapy. Then, neuroscience research uses music to investigate emotions, perceptual-action intermediaries, and social cognition, including illustrative correlations in these areas of music therapy [3]. There is evidence that music therapy can improve the mental health of patients with depression. Therefore, the possible mechanism of this complex intervention is studied, and it is considered that music therapy is partially effective, because active music production within the therapeutic framework provides patients with new opportunities for aesthetic, physical, and relational experiences [4]. Music therapy is a potential nondrug treatment for the behavioral and psychological symptoms of dementia, and while some studies have found it helpful, most are small and uncontrollable. Music therapy is a safe and effective method to treat anxiety and restlessness in patients with moderate and severe Alzheimer's disease. This is consistent with the results of some noncontrol studies on music therapy for dementia [5]. The field of brain-computer interface represents a more interesting field in neurophysiology research, because it studies the development of machines that transform the brain's “thoughts” into certain predefined behaviors. The research shows that the EEG data measured in complex dynamic visual motion tasks carry enough information about the current motion, which can be successfully extracted by appropriate signal processing and recognition methods [6]. The idea of brain-computer interface based on EEG is to help those who are unable to communicate ideas due to neuromuscular diseases and thus affected by motor disorders. Wavelet transform and other techniques are used to preprocess the data, and linear predictive coding is used to determine autoregressive coefficients as feature vectors, and neural networks are trained for classification. Then, the data of 140 random experiments are tested on the trained network, and the efficiency of this method is determined to be 71.5% [7]. The application of steady-state visual evoked potential (SSVEP) in brain-computer interface (BCI) system has attracted more and more attention. An online multichannel brain-computer interface system based on SSVEP is proposed, which uses canonical correlation analysis (CCA) to extract frequency information related to SSVEP. Experimental results show that the BCI system has high performance, with an average accuracy of 95.3% [8]. People can learn to control the EEG characteristics composed of sensorimotor rhythm amplitudes and can use this control to move the cursor to the target on the screen in one or two dimensions. The results show that the order selection of autoregressive model is an important determinant of BCI performance, which should be based on the criteria reflecting system performance [9]. A time-frequency (TF) method for extracting features from electroencephalogram (EEG) images of left and right hand movements is studied in this paper. Feature extraction process (FEP) extracts frequency domain information to form features, and at the same time, time-frequency resolution is obtained by localizing the fast Fourier transform (FFTs) of the signal to a specific window of time localization. This method is quantified by classification accuracy (CA), information transmission rate (IT), and mutual information (MI) and achieves good performance [10]. Common space mode (CSP) is one of the most widely used methods in brain-computer interface (BCI), which can enhance the separability of multichannel electroencephalogram (EEG) and other brain signals. This paper proposes to divide each class into many subclasses and describes this problem in a redesigned graph embedding framework with vertices as cluster centers. We have also redefined the traditional FLDA in our diagram embedding framework, which is helpful to develop and understand the proposed method. Experimental results show the superiority of this method [11]. Whether successful antidepressant therapy is associated with changes in psycho-behavioral strategies used to regulate mood is unclear. We examined depressive symptoms and emotion regulation strategies before and after antidepressants. Since we evaluated acute outcomes, it is not clear whether the effects of antidepressants on mood regulation will persist over time [12]. As we all know, serotonin can regulate mood, sleep, and appetite systematically, so it is related to the control of many behaviors and physiological functions. This paper reviews the latest progress in this field and discusses the mechanism of antidepressant acting on this target and its possible interaction with other components of serotoninergic neurotransmission [13]. Emotional regulation and impulse are the core aspects of borderline personality disorder (BPD) pathology. Although these two problems may be particularly combined in BPD, so far, few studies have studied impulsive emotion regulation in BPD. The results of this study are consistent with the view that the disorder of amygdala-prefrontal neural network in BPD patients is compensated by the subcortical loop involving subthalamic nucleus, which leads to the inhibition of normal behavior in these patients [14]. There is a great deal of evidence that stress response and stress adaptation dysfunction are in the pathophysiological mechanism of human depression (MDD). Endogenous opioid neurotransmission activates mu-opioid receptors to participate in stress and emotion regulation and is further related to MDD [15].

The article "Study on Antidepressant Emotion Regulation Based on Feedback Analysis of Music Therapy with Brain-Computer Interface" was published in 2022. Journal: Comput Math Methods Med.

## 2. Music Therapy

### 2.1. Mechanism of Music Therapy

Music therapy is a process of healing wounds, regulating emotions and physical functions by using melody, rhythm, and unique language and movements of music. In the limbic system, the amygdala is the central hub of neural circuit, which is deeply involved in the initiation, generation, detection, maintenance, regulation, and termination of emotions. Among them, blood level-dependent fMRI signals were relatively enhanced in ventral striatum and anterior insular lobe, while the amygdala, hippocampus, parahippocampal gyrus, and temporal polar region were relatively enhanced in musician's happy music stimulation. The fMRI-dependent signals from the amygdala, hippocampus, parahippocampal gyrus, and temporal polar regions were proportionally enhanced by randomly played discordant musical stimuli. These findings indicate that the center near the hippocampus plays an important role in the processing of acoustic roughness.

Balli et al.'s music research reveals for the first time that different regions of human amygdala have different functional characteristics in response to musical stimuli. In this study, harmonic piano music and sharp piano music were used as positive and negative stimuli, respectively, and the effects of two types of music on the dependence intensity of blood samples in the amygdala were examined. The results showed that under two different types of music stimulation, the dependent signal of blood samples in basolateral region increased, while the level-dependent signal of blood samples on amygdala surface decreased. The sample was weakened and the level-dependent signal from the blood sample was amplified in the superficial region of the amygdala. The functional network between brain structures involved in emotional processing is shown in Figure 1.

### 2.2. Social Functions of Music

Society is a living space where people can maintain each other and live together for a long time. People constantly participate in various social functions, and music activities are one of the comprehensive functions involving various social functions.

The early form of music is to express personal communication information through sound level and volume. With the development of human society, music activities greatly enrich the ways and means of expressing emotions, and people also integrate national culture and social environment into music. The reason why music can evolve from simple thought expression to contemporary music functions such as concert, recital, and drama is the result of the interaction between music and society. Examples of the influence of music creation on social individuals include the following:

Close communication of thoughts and emotions strengthens social skills, builds mutual trust, and effectively prevents social isolation. Compared with traditional medical methods, it is more helpful to cure mental diseases. Therefore, involving depressed patients in making music is usually more beneficial to treat depression than listening to music, because it can improve expression and communication skills, improve social relations, and prevent social isolation of depressed patients. In addition, making music involves changes in social cognitive skills. Social cognition is a process of analyzing and understanding the external environment.

The article "Study on Antidepressant Emotion Regulation Based on Feedback Analysis of Music Therapy with Brain-Computer Interface" was published in 2022. Journal: Comput Math Methods Med.

In a word, different music activities are often accompanied by changes in different social activities. These social activities can affect the external performance of depressed patients, for example, improve social skills, improve emotional state, and improve cognitive level. This provides theoretical support for the follow-up use of music activities as a means to regulate depression.

### 2.3. Methods of Music Therapy Feedback to Regulate Depression

According to the above theoretical knowledge, this paper proposes a brain-computer interface music therapy feedback analysis of depression emotion regulation method. The flow is shown in Figure 2.

Long-term depression is the main symptom of depression. When patients with depression are stimulated by external pressure, they will process the stimulus through the structure of limbic system and produce corresponding negative emotions. One way to regulate depression through music feedback is to use EEG signals to monitor patients' emotions and convert this signal into music signals that patients can understand.

## 3. Algorithm of EEG Signal Processing by CNN

### 3.1. Basic Network of Convolution Neural Network

CNN network is an important part of deep learning algorithm research. Its essence can be regarded as an artificial neural network that transmits feedback, inspired by the abstract process of human vision. Every neuron in CNN network can be considered as a neuron corresponding to human visual field, which is simulated and does not need much manual processing to train. The CNN model is not as popular as it used to be in the EEG classification of movie tasks. A very important reason is that until now, it is difficult to find an effective transformation method to represent EEG signals, so that the EEG shape of signals can better match the way CNN processes data.  Figure 3 shows the basic structure of CNN network.

As shown in Figure 3, the basic structure of CNN network is mainly composed of input layer, convolution layer, pooling layer, FC layer, and other network structure layers.

The article "Study on Antidepressant Emotion Regulation Based on Feedback Analysis of Music Therapy with Brain-Computer Interface" was published in 2022. Journal: Comput Math Methods Med.

The important network layers are explained below.

#### 3.1.1. Convolution Layer

Convolution layer is related to the performance of the whole network when assembling and decomposing data. The convolution calculation of the input data of the previous layer through convolution adjustment is essentially a weight matrix, and the characteristics of the convolution layer can be finally determined after the offset value is processed by a certain trigger function.

Convolution transport can be expressed mathematically by

(1) $$\begin{array}{c} k*g=\int_{-\infty }^{+\infty }k\left(\tau \right)g\left(\tau -t\right)dt. \end{array}$$

In this way, the convolution editing process of convolution layer can be expressed as

(2) $$\begin{array}{c} C_{j}^{L}=f\left(\underset{i\in N^{L-1}}{\sum }C_{i}^{L-1}*W_{j}^{L}+b_{j}^{L}\right), \end{array}$$

where *C*_*j*_^*L*^ represents the *J*th feature map of the *L*th convolution layer, *C*_*i*_^*L*−1^ represents the *L* − 1 layer, that is, the feature map of the previous layer, which is also the input of the *L*th layer, and *W*_*j*_^*L*^ is the feature layer of the *J*th layer.

It should be noted that the connection weights between different neurons on the same layer are universal, so this design is beneficial to the convergence of the model. In order to improve the performance of network architecture, functions such as ReLU, sigmoid, and tanh are often used. Formulas (3), (4), and (5), respectively, express different mathematical expressions of the above joint activation function:

(3) ReLU:fx=max0,x,

(4) $$\begin{array}{c} \text{sigmoid}:f\left(x\right)=\frac{1}{1+e^{-x}}, \end{array}$$

(5) $$\begin{array}{c} \tanh:f\left(x\right)=\frac{1-e^{-2x}}{1+e^{-2x}}. \end{array}$$

#### 3.1.2. Pooling Layer

The neurons in the pooling layer are the same as those in the convolution layer. Generally speaking, there are two commonly used pooling methods: maximum pooling and average pooling. For comparison, the maximum value is selected as the output of this range, and the merging process can be simplified to

(6) $$\begin{array}{c} P_{j}^{K}=\text{down}=\left(\underset{i\in N^{K-1}}{\sum }C_{i}^{K}\beta_{j}^{K}+b_{j}^{K}\right), \end{array}$$

where *P*_*j*_^*K*^ represents the *J*th feature map of the *K*th pooled layer, *β*_*j*_^*K*^ is the multiplier deviation of the *J*th pooled core of the *K*th layer, *b*_*j*_^*K*^ is the corresponding additional deviation, and down(·) represents different collections.

Generally, convolution layer and pooling layer appear alternately. As shown in Figure 4, the data set is represented by convolution layer with convolution size of 2 × 2 and pooling layer with size of 2 × 2. Examples of average pooling and maximum pooling are given.

The article "Study on Antidepressant Emotion Regulation Based on Feedback Analysis of Music Therapy with Brain-Computer Interface" was published in 2022. Journal: Comput Math Methods Med.

#### 3.1.3. Full Connection Layer

Generally speaking, the whole CNN network has one or more FC layers. At present, the activation functions commonly used in FC layers are ReLU and sigmoid.

### 3.2. EEG Classification Model Based on CNN Network

#### 3.2.1. Network Topology

In this section, we build a multilayer network model to analyze data. The whole identification process is shown in Figure 5.

*(1) Build a CNN Model for ECoG Data*. The CNN model structure is shown in Figure 6.

Input layer: in the input layer, each original signal is a tensor matrix, and the sample data is transformed into a tensor matrix with dimension [*N*_*e*_, *N*_*s*_, 1], so that EEG data can be regarded as gray images, which is

(7) $$\begin{array}{c} a_{j}^{0}\left(m\right)=x_{i}\left(m\right), \end{array}$$

wherein *x*_*i*_(*m*) represents the data of the *m*th sampling point of the *i*th electrode channel, 1 ≤ *i* ≤ *N*_*e*_, 1 ≤ *m* ≤ *N*_*s*_.

Conv1 layer: according to the characteristics of convolution layer, ECoG data is processed by

(8) ajLm=ReLU∑i=1NsaiL−1m∗WjL−1m+bjL−1,

where *L* is the number of convolution layers, there are four convolution layers, and each convolution layer is followed by a pooling layer.

Pool 1 layer: it can speed up the processing speed of the algorithm without losing data, and the calculation formula is shown in

(9) $$\begin{array}{c} a_{j}^{\left(K\right)}\left(m\right)=\max\left(\overset{N_{e}}{\underset{i=1}{\sum }}a_{i}^{\left(K-1\right)}\left(m\right)\cdot \beta_{j}^{\left(L-1\right)}\left(m\right)+b_{j}^{K}\right), \end{array}$$

where *K* is the number of pooled layers and there are four pooled layers, so the values of *K* are 2, 4, 6, and 8. *β*_*j*_^*K*^ is the coefficient bias and *b*_*j*_^*K*^ is the additional bias.

FC1: FC1 is the first fully connected layer to properly increase network depth.

Output layer: the output layer can use softmax function to classify the previously extracted high-level data, and the calculation expression is shown in

(10) $$\begin{array}{c} a^{\left(11\right)}=\text{soft}\max\left(\overset{N_{s}}{\underset{i}{\sum }}a^{\left(10\right)}W^{\left(11\right)}+b^{\left(11\right)}\right). \end{array}$$

The expression for softmax is shown in

(11) $$\begin{array}{c} \text{soft}\max\left(x_{i}\right)=\frac{e^{x_{i}}}{\sum_{n=1}^{N}e^{x_{n}}}. \end{array}$$

Finally, a vector *a*^(11)^ = [*a*_0_^(11)^, *a*_1_^(11)^]^*T*^ is output, *a*_0_^(11)^ represents the probability of belonging to a fictitious task, and *a*_1_^(11)^ represents the probability of not belonging to a fictitious task.

*(2) Constructing CNN Model from EEG Data*. The CNN network topology based on EEG data is similar to the network topology based on ECoGEEG signal. The difference is that the number of network layers used is different.

The article "Study on Antidepressant Emotion Regulation Based on Feedback Analysis of Music Therapy with Brain-Computer Interface" was published in 2022. Journal: Comput Math Methods Med.

It should be noted that in order to improve the efficiency of the algorithm, Dropout and L1 adjustment are also used to prevent overfitting as much as possible. In order to promote the complex cooperation between neurons and improve the learning ability of the model, the weights of neurons are randomly reset with a certain probability. The above two methods are widely used in neural network training to reduce overfitting. This article is also based on CNN mechanism to suppress the influence of overfitting.

#### 3.2.2. Network Parameter Training

The CNN model is based on ECoG and EEG-EEG data. As you can see from the previous section, using the input data vector *x*, the output of the model is *a*^(11)^ = [*a*_0_^(11)^, *a*_1_^(11)^]^*T*^, where *a*_*i*_^(11)^ represents the prediction probability of each class, giving a new result. If the actual title of the sample is *y* = [*y*_0_, *y*_1_]^*T*^, then when *N* samples are taught, the loss function is shown in

(12) $$\begin{array}{c} E=-\frac{1}{N}\overset{N}{\underset{n=1}{\sum }}\overset{1}{\underset{i=1}{\sum }}y_{i}\log\left(a_{i}^{\left(11\right)}\right). \end{array}$$

The formulas for calculating the weights and deviation gradients of the network are shown in

(13) $$\begin{array}{c} \frac{\partial E}{\partial W^{\left(11\right)}}=-\frac{1}{N}\overset{N}{\underset{n=1}{\sum }}\left[\frac{y_{0}}{a_{0}^{\left(11\right)}}\frac{\partial a_{0}^{\left(11\right)}}{\partial W^{\left(l\right)}}+\frac{y_{1}}{a_{1}^{\left(11\right)}}\frac{\partial a_{1}^{\left(11\right)}}{\partial W^{\left(l\right)}}\right], \end{array}$$

(14) $$\begin{array}{c} \frac{\partial E}{\partial b^{\left(l\right)}}=-\frac{1}{N}\overset{N}{\underset{n=1}{\sum }}\left[\frac{y_{0}}{a_{0}^{\left(11\right)}}\frac{\partial a_{0}^{\left(11\right)}}{\partial b^{\left(l\right)}}+\frac{y_{1}}{a_{1}^{\left(11\right)}}\frac{\partial a_{1}^{\left(11\right)}}{\partial b^{\left(l\right)}}\right]. \end{array}$$

Once the gradient is obtained, the parameters are updated according to the gradient descent method, as shown in

(15) $$\begin{array}{c} W_{t+1}=W_{t}-\eta \frac{\partial E\left(W,b\right)}{\partial W_{t}}, \end{array}$$

(16) $$\begin{array}{c} b_{t+1}=b_{t}-\eta \frac{\partial E\left(W,b\right)}{\partial b_{t}}. \end{array}$$

High speed means that it takes less time for the model to reach the convergence point. At high speed, the model jumps too much and cannot find the optimal center of gravity.

#### 3.2.3. Classification Algorithm

As a machine learning algorithm, GB classifier is used to get a strong classifier from many classifications. Its basic idea is to continuously optimize the loss function of the model in order to obtain stronger prediction or classification ability. The power of the model is constantly increasing. According to mathematical theory, when the loss function follows the direction of its data gradient, it can achieve the best and fastest decline.

The article "Study on Antidepressant Emotion Regulation Based on Feedback Analysis of Music Therapy with Brain-Computer Interface" was published in 2022. Journal: Comput Math Methods Med.

If the function data performed by the CNN network is *o*_*i*_, the mathematical representation is shown in

(17) $$\begin{array}{c} L\left(F_{m};O;Y\right)=\log\left(\overset{N}{\underset{i=1}{\prod }}p_{m}{\left(y_{i}=1\left|o_{i}\right.\right)}^{y_{i}}p_{m}{\left(y_{i}=0\left|o_{i}\right.\right)}^{1-y_{i}}\right), \end{array}$$

where the logarithmic regression model is defined as shown in

(18) $$\begin{array}{c} p_{m}\left(y_{i}=1\left|o_{i}\right.\right)=\frac{e^{F_{m}\left(o_{i}\right)}}{e^{F_{m}\left(o_{i}\right)}+e^{-F_{m}\left(o_{i}\right)}}. \end{array}$$

The initial value of logarithmic regression model is preset as *p*_0_(*y*_*i*_ = 1|*o*_*i*_) = 0.5.

Taking ordinary least square regression as the minimum loss function, GB algorithm based on OLS regression can be expressed as the following process:

1. Calculate the gradient of the loss function in the direction of gradient descent, as shown in

(19) $$\begin{array}{c} {\bar{y}}_{i}={\left[\frac{\partial L\left(F\left(o_{i}\right)\right)}{\partial F\left(o_{i}\right)}\right]}_{F=F_{m-1}}=2\left(y_{i}-p_{m-1}\left(y_{i}=1\left|o_{i}\right.\right)\right) \end{array}$$

(2) Based on the OLS, select the appropriate gradient, as shown in

(20) $$\begin{array}{c} f_{m}=\arg\underset{f}{\min}\overset{N}{\underset{i=1}{\sum }}{\left(\bar{y}-f\left(o_{i}\right)\right)}^{2} \end{array}$$

The result of the weak classifier is that the vector *o*_*i*_(*t*) of the EKoG sample is projected onto the regression coefficient *a* at time *t*, as shown by

(21) $$\begin{array}{c} f\left(o_{i},a,t\right)=a^{T}o_{i}\left(t\right). \end{array}$$

(*a*_*m*_, *t*_*m*_) when the error is minimized, it is then selected as the parameter of the weak classification, as shown by

(22) $$\begin{array}{c} f_{m}\left(o_{i}\right)=f\left(o_{i},a,t\right). \end{array}$$

(3) Then, calculate its weight, as shown in

(23) $$\begin{array}{c} \gamma_{m}=\arg\underset{\gamma }{\max}L\left(F_{m-1}+\gamma f_{m};O,Y\right) \end{array}$$

(4) Multiply a small number *ε* in each step, reduce the value of *γ*_*m*_, and then get a strong classification through iteration, which can improve the generalization ability of the algorithm as shown in

(24) $$\begin{array}{c} F_{m}=F_{m-1}+{\varepsilon \gamma }_{m}f_{m} \end{array}$$

(5) Finally, a new logarithmic regression value is obtained, as shown in

(25) $$\begin{array}{c} p_{m}\left(y_{i}=1\left|o_{i}\right.\right)=\frac{e^{F_{m}\left(o_{i}\right)}}{e^{F_{m}\left(o_{i}\right)}+e^{-F_{m}\left(o_{i}\right)}} \end{array}$$

Among them, in order to find the optimal iteration times and achieve fast classification, we use logarithmic regression model, which is not limited by the predicted value of the model.

The article "Study on Antidepressant Emotion Regulation Based on Feedback Analysis of Music Therapy with Brain-Computer Interface" was published in 2022. Journal: Comput Math Methods Med.

## 4. Experimental Research and Analysis

### 4.1. Selection of Preprocessing Algorithm for EEG Signal

In the preprocessing of EEG signal, there are short-time Fourier transform, wavelet transform, Gunner distribution, EMD, and other methods. In order to process the signal more intuitively and efficiently, we compare these algorithms in self-adaptation, high-efficiency deep mining ability of data and decomposition signal. Five comparative experiments are carried out, and the results are shown in Figures 7, 8, and 9.

Looking at the figure above, we can see that in the aspect of self-adaptation, the performance of data efficient deep mining ability and signal decomposition ability is compared. EMD algorithm has more advantages, so we can draw that EMD algorithm is intuitive, efficient, self-adaptive, hindsight, and other advantages.

### 4.2. Optimal Selection of Pretreatment Methods

This section describes SNIR, average energy, and MAPE to measure the system's ability to suppress noise. See formula (26) for SNIR calculation formula:

(26) $$\begin{array}{c} \text{SNIR}=\frac{{\text{SNR}}_{o}}{{\text{SNR}}_{i}}, \end{array}$$

where SNR_*o*_ is the signal-to-noise ratio of the system output and SNR_*i*_ is the signal-to-noise ratio of the system input. SNR is the average power ratio of signal to noise. The calculation formula is shown in

(27) $$\begin{array}{c} \text{SNR}=\frac{S}{N}. \end{array}$$

In decibels (dB), as shown in

(28) $$\begin{array}{c} \text{SNR}\left(\text{dB}\right)=10\times \log_{10}\left(\frac{S}{N}\right)\left(\text{dB}\right). \end{array}$$

The calculation formula of energy mean value is shown in

(29) $$\begin{array}{c} \bar{E}=\frac{1}{n}\overset{n}{\underset{i=1}{\sum }}x^{2}\left(i\right), \end{array}$$

where *x*(*i*) is the discrete amplitude of EEG signal after noise suppression and *N* is the number of sampling points.

The calculation formula for MAPE is shown in

(30) $$\begin{array}{c} M=\overset{n}{\underset{t=1}{\sum }}\left|\frac{A_{t}-F_{t}}{A_{t}}\right|\times \frac{100\%}{n}. \end{array}$$

Among them, the smaller the MAPE, the smaller the error.

SNIR, energy average, and MAPE are calculated for the original EEG signal after the above-mentioned “tenfold reduction” by three denoising methods, and the results are shown in Table 1.

The article "Study on Antidepressant Emotion Regulation Based on Feedback Analysis of Music Therapy with Brain-Computer Interface" was published in 2022. Journal: Comput Math Methods Med.

Table 2 shows the comparison results of Deap data set and self-collected data set, including 1152 EEG signal data sets, which have been processed by three noise reduction methods. Due to the large amount of data, the results are presented in the form of data sets.

In Table 1, the results show that EMD+FastICA algorithm has the highest SNIR, the lowest MAPE, and the lowest average energy value of EEG signals. Table 2 also clearly shows that better results can be obtained by mute calculation of three indexes for EEG signal data through EMD+FastICA algorithm.

### 4.3. Subjects

All the subjects selected in this experiment are graduate students. Four, eight, and four graduate students were selected as normal control group, depression control group, and feedback training group. Evaluation and feedback training are conducted once a week for a total of six weeks. The initial grouping criteria are shown in Table 3.

### 4.4. Experimental Flow

In order to make the experimental results more accurate, our test site was chosen in a relatively undisturbed room. And the test time is strictly controlled within 45 minutes. The specific experimental process is as follows:

1. Rating stage scale: before each test, the user asked the subjects to complete three scales, SCL-90, SDS, and PHQ-9, so that the subjects could evaluate the degree of depression before the test. This step takes about 10 minutes
2. Experimental preparation stage: first, determine whether the subject can complete the test. After that, the operator explains the working principle of the system to the subject, feeds back the test process, matters needing attention in the test process, etc. Finally, the operator sticks electrode stickers on the positions of FP1, FP2, and FPZ electrodes on the forehead to ensure the normal acquisition of EEG signals. This step takes about 3 minutes

The feedback exercise stage includes one breathing exercise and two feedback exercises. Before the feedback training, the operator organized the subjects to practice breathing for 3 minutes. The purpose of this is to help the subjects relax and concentrate, so that the subjects can quickly adapt to feedback training. After that, the instructor guided the subjects through a series of two feedback exercises, each lasting 13 minutes. This step takes about 29 minutes.

(3) Training stage: in the previous article, we designed two feedback training methods: breathing and music. The specific feedback training process is shown in Figure 10
(4) Communication stage: in this stage, the experimenter communicates with the tester to understand whether the feedback music is effective and check whether the subjects can manage their physical condition skillfully. At the same time, the subjects are encouraged to listen to sober and exciting music when they are depressed and adjust their emotions through feedback training

The article "Study on Antidepressant Emotion Regulation Based on Feedback Analysis of Music Therapy with Brain-Computer Interface" was published in 2022. Journal: Comput Math Methods Med.

### 4.5. Statistical Analysis

#### 4.5.1. Scoring Analysis of Scale

Three scales, SCL-90, SDS, and PHQ-9, were selected to measure the degree of symptoms. Patient health questionnaire is used in the study. See Table 4 for the criteria of patients with depression. During the 6-week follow-up test, we selected the data measured at the first time as the baseline data.

SCL-90, SDS, and PHQ-9 were averaged among the three groups, and independent *T*-test was performed. The results are shown in Tables 5, 6, and 7. It can be seen from the table that before feedback training, there is little difference in scale scores between the feedback training group and depression control group. With the progress of feedback training, the difference between the feedback training group and the depression control group became larger and larger. In the sixth test evaluated by SDS and PHQ-9, it was found that there were significant differences between the feedback training group and some correlations between the normal controls. Obviously, the method designed in this paper can effectively improve the condition of patients with mild depression.

Figures 11, 12, and 13 show the changes in the scores of the three corresponding SCL-90, SDS, and PHQ-9 scales over a six-week period. It can be observed that the scale evaluation scores of the feedback training group showed a downward trend, indicating that music feedback has a positive effect on emotional regulation. When the two control groups did not participate in feedback training, the scores of individual subjects were different, and there was no obvious trend in the overall scale scores. In addition, with the passage of time, the evaluation scores in the feedback training group decreased more and more obviously, especially in the third to sixth tests. This shows that the emotion regulation method with music feedback proposed in this paper is always effective in regulating the depression of patients with mild depression. At the same time, after the first three music feedback experiments, the negative emotions were improved, and the performance was further improved with the help. Music regulates itself. During the follow-up period, emotional regulation and depressive symptoms improved.

In addition, because the subjects of this study are educated graduate students, during the experiment, the subjects are more or less aware of the treatment of depression and receive some degree of cognitive behavioral therapy. This may also be the reason why the subjects can quickly adapt to music therapy and adjust themselves in the experiment.

The article "Study on Antidepressant Emotion Regulation Based on Feedback Analysis of Music Therapy with Brain-Computer Interface" was published in 2022. Journal: Comput Math Methods Med.

#### 4.5.2. Quantity Analysis of Emotional Fragments

This paper also analyzes the changes of emotional fragments of EEG signals in music experiments. The EEG character sequences obtained by us are divided into three types: active state, passive state, and normal state. The length of each type of EEG character sequence is 0.5 s. For each music feedback test, we conducted two feedback trainings. For each music feedback test, we need to calculate the emotional state within 6 seconds. During the experiment, the system needs to convert 399 segments, about 4788 EEG markers. Among them, the number of strings in each EEG signal is too much, which is not intuitive. Therefore, this section selects the feedback music segments that change during the experiment to reflect the changes of subjects' emotions.

The change trend of the number of feedback music segments in the feedback training group is shown in Figure 14. Observation shows that feedback music representing positive emotions is increasing. Among them, the changes of feedback music fragments from the first trial to the third trial are obviously different from those from the third trial to the sixth trial. The reason may be that during the first and third experiments, the emotional state of the subjects changed from negative to normal due to music feedback training. Therefore, the number of music fragments representing negative emotions first decreased and then increased slowly, while the number of music fragments representing positive emotions first increased slowly and then increased rapidly.

In the experiment of converting EEG into music, the signal sequence of EEG signals obtained by music stimulation will be affected by the characteristics of depressed patients. The test strictly screens the characteristics of depressed patients such as age, education level, and medical history, so the application range of EEG signal feature set obtained in the test is limited. In addition, in the EEG conversion music experiment, there are only three kinds of music stimuli (positive, medium, and negative), so there is less emotional feedback. Future research should consider the differences of different target groups and individual knowledge and increase the types of music stimulation in the experiment, so that the system can be applied to the treatment of a wider range of mental health disorders.

## 5. Concluding Remarks

Depression has become a very common disease in people's daily life. Modern people are under increasing pressure in life, work, and study. Contradictions and setbacks make people exhausted. Music therapy is a new interdisciplinary subject, which combines the essence of music, medicine, and psychology. It is a process in which music therapists help patients break through psychological barriers and recover their physical and mental health through specially designed music models. Music therapy is mainly based on the theory and method of psychotherapy, which makes use of the unique psychological and physiological effects of music. The results of this study show that the quality of life and anxiety symptoms of depressed patients have been improved after music therapy, especially music therapy combined with EEG feedback training. If it can be popularized in the treatment of depressed patients, it will be a great boon for patients.

The article "Study on Antidepressant Emotion Regulation Based on Feedback Analysis of Music Therapy with Brain-Computer Interface" was published in 2022. Journal: Comput Math Methods Med.

## Figures and Tables

**Figure 1:** Functional network diagram of brain structure involved in emotional processing.

**Figure 2:** Description diagram of music feedback control method for depression based on EEG.

**Figure 3:** Basic structure diagram of CNN network.

**Figure 4:** Example of convolution and pooling.

**Figure 5:** Flow chart of moving image classification task recognition based on CNN model.

**Figure 6:** Network topology diagram of CNN.

**Figure 7:** Comparison of adaptability.

**Figure 8:** Comparison of signal decomposition ability.

**Figure 9:** Comparison of data mining capabilities.

**Figure 10:** Flow chart of feedback training.

**Figure 11:** The change trend of SCL-90 scale score.

**Figure 12:** Change trend of SDS scale score.

**Figure 13:** Change trend of PHQ-9 scale score.

**Figure 14:** The change trend of the number of feedback music clips corresponding to positive and negative emotions.

**Table 1:** Three noise reduction methods.

EEG signal classification	SNIR (dB)	Average energy (*μ*V)	MAPE (%)
After EMD algorithm denoising	-4.5609	1.2826	2.3974
After denoising by FastICA algorithm	-3.6278	0.977	1.9444
After EMD+FastICA algorithm denoising	0.1866	0.6227	1.5044

**Table 2:** Comparison of denoising effects of three methods based on all EEG data.

EEG signal classification	SNIR (dB)	Average energy (*μ*V)	MAPE (%)
After EMD algorithm denoising	−4.5039 ± 0.6057	1.4549 ± 0.1447	2.4473 ± 0.5843
After denoising by FastICA algorithm	−2.9835 ± 0.9539	1.1311 ± 0.1781	1.7389 ± 0.6545
After EMD+FastICA algorithm denoising	1.0123 ± 0.2012	0.7501 ± 0.2398	1.1326 ± 0.3794

**Table 3:** Subject grouping criteria.

Group name	SCL-90 score	SDS score	PHQ-9 score	Feedback training times	Scale evaluation times
Normal control group	<8	<53	<5	0	6
Depression control group	>26	53-62	5-9	0	6
Feedback training group	>26	53-62	5-9	6	6

**Table 4:** Scoring standards of SCL-90, SDS, and PHQ-9.

Degree of depression	SCL-90	SDS	PHQ-9
Normal	0-26	0-52	0-4
Mild	>26	53-62	5-9
Moderate		63-72	10-14
Moderate and severe		>72	15-29
Severe			20-27

The article "Study on Antidepressant Emotion Regulation Based on Feedback Analysis of Music Therapy with Brain-Computer Interface" was published in 2022. Journal: Comput Math Methods Med.

**Table 5:** SCL-90 scale evaluation statistics.

Mean and standard deviation of SCL-90 scale				*T*-test		
Number of experiments	Feedback training group I	Depression control group II	Normal control group III	I and II	I and III	II and III
Baseline	31.40 ± 5.10	31.53 ± 5.66	2.74 ± 3.19	0.9482	0.0000	0.0000
2	29.75 ± 2.33	31.83 ± 6.30	2.37 ± 2.96	0.4065	0.0000	0.0000
3	28.04 ± 1.60	31.14 ± 4.52	2.75 ± 3.18	0.0025	0.0000	0.0000
4	24.30 ± 1.75	31.23 ± 5.09	2.60 ± 3.16	0.0000	0.0000	0.0000
6	17.20 ± 2.87	30.82 ± 3.16	2.12 ± 2.12	0.0000	0.0000	0.0000

**Table 6:** Evaluation statistics of SDS scale.

Mean and standard deviation of SDS scale				*T*-test		
Number of experiments	Feedback training group I	Depression control group II	Normal control group III	I and II	I and III	II and III
Baseline	56.75 ± 2.41	56.77 ± 2.58	34.37 ± 5.92	0.9703	0.0000	0.0000
2	55.42 ± 2.48	56.42 ± 2.12	33.91 ± 5.72	0.1734	0.0000	0.0000
3	50.59 ± 3.57	56.64 ± 2.55	34.00 ± 5.93	0.0000	0.0000	0.0000
4	46.50 ± 2.14	56.79 ± 2.54	34.19 ± 5.75	0.0000	0.0000	0.0000
6	37.54 ± 5.79	56.30 ± 2.58	34.30 ± 5.91	0.0000	0.0742	0.0000

**Table 7:** Evaluation statistics of PHQ-9 scale.

Mean and standard deviation of PHQ-9 scale				*T*-test		
Number of experiments	Feedback training group I	Depression control group II	Normal control group III	I and II	I and III	II and III
Baseline	6.37 ± 1.09	6.38 ± 1.26	1.25 ± 1.37	0.9580	0.0000	0.0000
2	6.00 ± 1.22	6.39 ± 1.21	1.27 ± 1.36	0.1923	0.0000	0.0000
3	4.72 ± 1.59	6.39 ± 1.33	1.29 ± 1.38	0.0000	0.0000	0.0000
4	3.79 ± 0.80	6.44 ± 1.14	1.14 ± 1.31	0.0000	0.0000	0.0000
6	2.24 ± 1.08	6.38 ± 1.21	1.25 ± 1.37	0.0000	0.0202	0.0000

## Data Availability

The experimental data used to support the findings of this study are available from the corresponding author upon request.
